# Urinary RBP as an Independent Predictor of Renal Outcome in Diabetic Nephropathy

**DOI:** 10.1155/2022/9687868

**Published:** 2022-10-17

**Authors:** Fanghao Cai, Li Zhang, Peng Zhao, Fengping Qiu, Abdullahi Mohamed Mukhtar, Yanhong Ma, Jianghua Chen, Fei Han

**Affiliations:** ^1^Kidney Disease Center, The First Affiliated Hospital, Zhejiang University School of Medicine; Institute of Nephrology, Zhejiang University; Key Laboratory of Kidney Disease Prevention and Control Technology, Zhejiang Province; Zhejiang Clinical Research Center of Kidney and Urinary System Disease, Hangzhou, China; ^2^Sanmen People's Hospital, Ningbo, China; ^3^Haining People's Hospital, Jiaxin, China; ^4^Huzhou First People's Hospital, Huzhou, China

## Abstract

**Background:**

Renal tubular impairment is prevalent in diabetic nephropathy (DN) and the histological severity predicted renal outcome. Biomarkers of tubular injury also increased in the urine of DN patients. The retrospective study aimed to assess the prognostic value of clinically widely applied urinary tubular injury markers, retinol-binding protein (RBP), *β*2-microglobulin (*β*2-MG) and N-acetyl-*β*-D-glucosaminidase (NAG) in DN.

**Method:**

A total of 305 patients with biopsy-proven DN were enrolled. The baseline urine total protein and components including albumin, IgG, RBP, *β*2-MG and NAG were retrieved from medical records. The primary outcome was end stage renal disease (ESRD). Cox proportional hazard analysis and restricted cubic splines were performed to evaluate the association of parameters with ESRD. Nomograms were constructed and concordance index (C-index) was used to measure the prediction ability.

**Result:**

The levels of urinary RBP, *β*2-MG and NAG were positively correlated with the severity of interstitial fibrosis and tubular atrophy (IFTA). Positive correlations were also observed among *β*2-MG, NAG and mesangial expansion. Urinary RBP was not correlated with any glomerular lesions. Urinary RBP, *β*2-MG and NAG were risk factors for ESRD in hazard analysis with adjustment for age, gender and body mass index (BMI). The hazard ratios increased with the increment of baseline levels. In the multivariate Cox model including serum creatinine (SCr), total urinary protein, urinary albumin, urinary IgG and the tubular injury biomarkers, urinary RBP (with every g/mol.Cr increase: HR 1.06, 95% CI 1.03-1.10, *p* =0.001) remained as an independent risk factor for ESRD in DN patients. Patients were divided by the medium value of urinary RBP into the low RBP and high RBP groups. Survival analysis showed that significantly more patients in the high RBP progressed to ESRD compared to those in the low RBP group (*p* =0.02) when urinary total protein was less than 3.5 g/g. The C-index of the nomogram incorporating age, gender, BMI, SCr and total urine protein was 0.757. The value increased to 0.777 after adding urinary RBP to the model.

**Conclusions:**

Urinary RBP excretion was only correlated with the severity of IFTA and independently predicted ESRD in DN patients.

## 1. Introduction

Diabetic nephropathy (DN) is a common but devastating complication of diabetes mellitus (DM). In the recent annual data report on kidney disease in China, diabetes was considered the cause of 26.70% of patients with chronic kidney disease (CKD) and presented in 33.14% of patients entering dialysis [1]. DN patients suffered inevitable deterioration of kidney function. Glomerular damage was used to be recognized as the dominant culprit of DN progression. In recent decades, mounting lines of evidence emphasized the importance of tubular damage in the pathogenesis and progression of DN. In renal pathology, tubular injury could occur early and was prevalent. And the severity of tubulointerstitial lesions correlated with renal outcomes [2]. In clinical research of large cohorts across countries, 6%-14% of diabetic patients with deteriorated renal function did not develop albuminuria [3–5]. The presence of uncoupling of urinary protein excretion and kidney function deterioration highlighted the clinical application of urinary tubular injury markers in DN monitoring.

Urinary tubular injury markers increased early and vastly in diabetic patients with CKD. Their increments were observed in patients with normal albuminuria and could be used as complementary measurements to albuminuria and estimated glomerular filtration rate (eGFR) in early diagnosis of diabetic kidney disease, defined by the presence of microalbuminuria or impaired renal function [6, 7]. In terms of prognostic value for renal failure, whether the addition of urinary tubular biomarkers to known promoters of progression could improve prognostication was controversial. A prospective study of patients with diabetic kidney disease showed that the urinary tubular markers, neutrophil gelatinase-associated lipocalin (NGAL), Cystatin C and kidney injury molecule-1 (KIM-1) could independently predict faster eGFR decline and end stage renal disease (ESRD) [8]. Another ancillary study of a randomized clinical trial demonstrated that urinary retinol-binding protein (RBP) and monocyte chemoattractant protein-1 (MCP-1) were independently related to the risk of doubling of serum creatinine (SCr) or death in diabetic patients with macroalbuminuria [9]. But two studies of diabetic patients with proteinuria and diabetic patients with biopsy-proven DN, respectively, demonstrated that urinary NGAL, KIM-1 and *β*2-microglobulin (*β*2-MG) did not predict ESRD independent of the known promoters [10, 11]. The inconsistent findings might be due to discrepancies in different tubular injury markers, a small number of populations, and heterogeneity of enrolled patients. Subjects were of different urinary total protein levels, and the percentage of patients who developed CKD resulting from hypertension, obesity, ischemia, aging-related nephron loss, diabetic glomerular atherosclerosis or tubulointerstitial impairment was unclear [12]. So there need more studies to verify the predictive implication of urinary tubular injury biomarkers. And participants with renal pathological findings would help more accurately interpret the application. But studies evaluating tubular injury biomarkers in DN patients with renal biopsy were limited.

The present study recruited a relatively large number of DN patients confirmed by renal biopsy. It aimed to investigate the prognostic value of three widely available urinary tubular biomarkers, i.e., RBP, *β*2-MG and N-acetyl-*β*-D-glucosaminidase (NAG), and their relationship with clinicopathological presentations.

## 2. Methods

### 2.1. Patients

The study was in compliance with the Declaration of Helsinki and approved by the Committee on Research Ethics of the First Affiliated Hospital Zhejiang University School of Medicine. Subjects with renal biopsy-proven DN from March 2011 to August 2020 in our center were retrospectively recruited for the study. The exclusion criteria were CKD 3 stage, acute kidney injury, concurrent primary or secondary glomerulonephritis, or hypertensive nephropathy. Patients with follow-up for less than 6 months were also excluded except for those who reached the endpoint.

### 2.2. Clinical Information

Data were retrieved from the medical record. Laboratory examinations including glycated hemoglobinA1c (HbA1c), hemoglobin, serum albumin, serum lipids, SCr, eGFR and urinary proteins within 1 week of renal biopsy were collected. Urinary protein to creatinine ratio was used to represent 24-h urine protein. Urinary albumin and urinary immunoglobin G (IgG) were used to reflect kidney glomerular impairment, and urinary RBP, *β*2-MG and NAG were to reflect tubular injury. The endpoint was defined as ESRD.

### 2.3. Detection of Urinary Biomarkers

First-morning urine samples were obtained for urinary tests. Total urinary protein was quantified by a pyrogallol red-molybdate method (Jiuzhoutaikang, Beijing, China). The concentrations of urinary albumin (Dialab, Vienna, Austria), IgG (DENUO, Shanghai, China), RBP (Zybio, Chongqing, China), and *β*2-MG (Zybio, Chongqing, China) were measured by an immunoturbidimetric method using commercial kits. Urinary NAG was measured using the 6-methyl-2-thiopyridine-N-acetyl-indole-D-glucosaminidase substrate method (Seaful, Beijing, China). The values of urinary biomarkers were expressed as the ratio of the concentration to the concurrent urinary creatinine levels.

### 2.4. Renal Pathology

Each biopsy specimen went through standard processing. Two pathologists reported the diagnosis and pathological features separately. The diagnosis and classification of DN were done according to the criteria of Tervaert et al. [13]. Class I was defined as glomerular basement membrane thicker than 395 nm in females and 430 nm in males with mild or nonspecific light microscopy changes. Class II was mild (Class IIa) or severe (Class IIb) mesangial expansion and did not meet the criteria of Class III or Class IV. Class III was the presence of nodular sclerosis and Class IV was more than 50% global glomerulosclerosis. Semiquantitative scores for glomerular, tubulointerstitial, and vascular lesions were as follows [13]. Mesangial expansion and interstitial fibrosis and tubular atrophy (IFTA) were measured as 0 for absent, 1 for <25%, 2 for 25–50%, and 3 for >50% of the observed mesangial or tubulointerstitial areas. Arteriolar hyalinosis was scored as 0 for absent, 1 for one area of arteriolar hyalinosis and 2 for more than one area of arteriolar hyalinosis.

### 2.5. Statistical Analysis

SPSS version 22.0 and R software version 4.1.0 were performed for statistical analyses. Quantitative variables were interpreted as the mean ± standard deviation or the median with an interquartile range. The differences were compared using Student's t-test or Mann–Whitney *U* test as appropriate. Categorical data were interpreted as counts and percentages, and the differences were analyzed using the Chi-square test. The pathological correlations to the biomarkers were calculated using the Spearman correlation coefficient. The association of a clinical indicator with renal survival time was analyzed using a univariate Cox proportional hazard regression model and restricted cubic spline while adjusting for age, sex and body mass index (BMI). Multivariable Cox proportional hazards regression models with forward LR were performed to find independent risk factors. Kaplan–Meier curves were used to analyze the outcomes. Nomogram prognostic model was constructed based on the results of multivariate Cox analysis. The predicted ability was measured by concordance index (c-index). *P* values <0.05 were considered significant.

## 3. Results

### 3.1. General Characteristics

A total of 305 DN patients were enrolled in the study (Figure 1), and 232 were male (76.1%). Their age was 52.71 ± 10.45 years. The duration of diabetes was 8.43 ± 6.21 years, and 152 of 231 patients (65.8%) had diabetic retinopathy. One hundred and thirty-nine (45.57%) patients had baseline eGFR of higher than 60 ml/min/1.73m^2^, and 120 (39.34%) patients were in CKD 3 Stage. Urinary RBP, *β*2-MG and NAG were increased in 95.74%, 89.51% and 89.05% patients, respectively. In renal pathology, tubulointerstitial impairment was prevalent. IFTA was observed in 99.34% of patients and graded as moderate or worse in 70.16% of the patients.

### 3.2. Urinary Tubular Markers with Pathological Correlations

The pathological relations were shown in Figure 2. There were significant positive correlations between the urinary tubular biomarkers and IFTA score (*ρ* =0.191, *p* =0.001 between RBP and IFTA score; *ρ* =0.355, *p* <0.001 between *β*2-MG and IFTA score, *ρ* =0.139, *p* =0.044 between NAG and IFTA score). Urinary RBP did not correlate with glomerular impairment such as DN glomerular classes or mesangial expansion. While urinary *β*2-MG and NAG excretion were also significantly correlated with mesangial expansion. All the tubular injury markers were not associated with arteriolar hyalinosis.

### 3.3. Tubular Injury Markers as Risk Factors for ESRD

Associations between urinary tubular injury markers and renal outcome were analyzed using Cox proportional hazard model and restricted cubic spine with adjustment for age, gender and BMI. Cox analysis suggested tubular injury markers of RBP (with every g/mol.Cr increase: HR 1.05, 95% CI 1.03-1.07, *p*<0.001), *β*2-MG (with every g/mol.Cr increase: HR 1.18, 95% CI 1.10-1.27, *p*<0.001) and NAG (with every U/mol.Cr increase: HR 1.20, 95% CI 1.09-1.30, *p*<0.001) were risk factors for ESRD (Table 1) and the renal failure risk increased with the increase of the baseline tubular injury markers (Figure 3).

To further assess the independent effect, indicators were further adjusted for SCr. Urinary RBP and NAG remained significant. In the multivariate Cox model, we pooled all the clinical laboratory urinary kidney injury molecular markers, kidney function and influential clinical characteristics including blood pressure, hemoglobin and lipid indexes which were selected by the above variance analysis. In this model, urinary RBP (with every g/mol.Cr increase: HR 1.06, 95% CI 1.03-1.10, *p* =0.001) remained significant as an independent risk factor for ESRD (Table 1). Besides, gender as male (HR 1.75, 95% CI 1.06-2.90, *p* =0.029), baseline urinary protein to creatinine ratio (with every g/g increase: HR 1.2, 95% CI 1.12-1.29, *p* <0.001), SCr (with every mg/dL increase: HR 2.29, 95% CI 1.73-3.04, *p* <0.001) were independent risk factors. BMI (with every kg/m^2^ increase: HR 0.92, 95% CI 0.87-0.97, *p* <0.010) and hemoglobulin (with every mg/dL increase: HR 0.88, 95% CI 0.79-0.98, *p* =0.017) were independent protective factors.

### 3.4. Clinical Features of Patients with Different Levels of Urinary RBP

As shown in Table 2, patients were divided by the medium value of urinary RBP into the low RBP (≤2.43 g/mol.Cr, n =152) and high RBP (>2.43 g/mol.Cr, n =153) groups. Demographically, there were more females in the high RBP group (*p* =0.007). Patients in the high RBP group demonstrated higher blood pressure, severer lipid disorder with significantly higher serum concentrations of total cholesterol (*p* =0.011), low-density lipoprotein cholesterol (LDL-C, *p* =0.006) and high-density lipoprotein cholesterol (HDL-C, *p* =0.006) levels compared to those in the low RBP group, even with similar prescription of antihypertension and lipid-lowering drugs. There was no difference in the diabetic duration, diabetic retinopathy percentage and HbA1c level between the groups.

Subjects in the high RBP group demonstrated significantly lower hemoglobulin (*p* =0.015), serum albumin (*p* <0.001), higher urinary total proteins (*p* <0.001), urinary albumin (*p* <0.001) and urinary IgG (*p* <0.001) excretion compared to those in the low RBP group. There was no significant difference in baseline eGFR or SCr between the groups.

### 3.5. Tubular Injury Biomarkers Predict ESRD

During the follow-up period of 22.73(13.15, 35.16) months, significantly more patients in the half of participants with high RBP levels progressed to ESRD (*p* <0.001, Figure 4). To assess the influence of urinary total protein on the relationship between the tubular injury markers and renal outcome, we separately analyzed patients with or without overt proteinuria. Among patients with overt proteinuria, survival curves of both RBP groups decreased steeply and the difference diminished. For patients with mild to moderate proteinuria, those with higher baseline RBP levels had significantly worse outcomes (*p* =0.022).

Further, we constructed nomogram models to predict renal outcome, and the prediction ability was measured by C-index. In our patients, the conventional model involving age, gender, BMI, SCr and total urine protein level had a C index of 0.757. Adding urinary RBP excretion to the model increased the C index to 0.777 (Figure 5).

## 4. Discussion

In the present cohort of 305 subjects with biopsy-proven DN, the vast majority demonstrated tubulointerstitial impairment and elevated urinary tubular injury markers. Among the three biomarkers we evaluated, *RBP and β2-MG are biomarkers of tubular dysfunction with low molecular weights of 21* kDa *and 11* kDa*, respectively. They can be freely filtered by glomeruli and almost fully reabsorbed by proximal tubules* [14]. NAG is a lysosomal hydrolase with a molecular weight of 150 kDa. Urinary NAG is only excreted by injured proximal tubular cells and the elevation reflects renal tubular structural damage [15]. A study of 210 patients with biopsy-proven DN showed urinary excretion of NAG and *β2-MG was correlated with IFTA score, but did not add prognostic value to the known indicators of urinary protein excretion and* eGFR [11]. Their results were consistent with ours. Our study additionally analyzed the histopathologic correlations and found that *urinary β*2-MG and NAG levels were also correlated with mesangial expansion. Their limited predictive value might be explained by the influence of glomerular damage or urine environment on measurement. *β*2-MG was unstable in acid urine, while RBP was reported to be a better alternative [14]. It was found that urinary RBP outperformed *β*2-MG to detect the impairment of proximal renal tubules in Fanconi Syndrom [16]. A study of 1053 diabetic patients assessing six urinary biomarkers including RBP and *β*2-MG found that urinary RBP yielded best diagnostic value for diabetic kidney disease [17]. In the present study, urinary RBP level was purely correlated with IFTA lesions and had independent prognostic value.

We explored the clinical characteristics of DN patients with high urinary RBP excretion. Their demographic feature was a higher proportion of females affected, different from that of DN glomerulopathy. Patients with higher urinary RBP levels manifested lower hemoglobulin than their lower RBP counterparts. This could be explained by endogenous erythropoietin production in the tubulointerstitial compartment of kidney, since higher urinary RBP level was related to severer tubulointerstitial damage. Notably, although patients with higher urinary RBP levels exhibited more serious tubular injury, the baseline kidney function was comparable to those with lower urinary RBP levels. And there was no significant association between urinary RBP excretion and DN glomerulopathy. Some clinical features of patients with high urinary RBP could hardly be explained by glomerular damage, which supported the perspective of tubulopathy in DN progression.

Patients with higher urinary RBP manifested dysregulation of cholesterol metabolism with higher levels of total cholesterol, LDL-C and HDL-C. Increased levels of cholesterol and LDL-C are linked to lipid accumulation and lipotoxicity in tissue. Heavy lipid droplet deposition is observed in renal tubules in DN and associated with tubular damage [18–20]. Uptake of cholesterol is increased by tubular epithelial cells in DN with downregulation of cholesterol efflux genes, e.g., ABCA1, ABCG and upregulation of lipoprotein receptors, e.g., LOX-1, CD36 [18, 21, 22], and aggravates oxidative stress in tubular epithelial cells. In addition, oxidized LDL could directly induce inflammation, apoptosis and fibrosis on tubular epithelial cells [23–25]. And oxidized LDL was reported able to predict eGFR deterioration in proteinuric diabetic kidney disease [23]. In our study, HDL-C levels concurrently increased. HDL-C is recognized as the good cholesterol, which can reverse cholesterol transport from peripheral tissues. Increased HDL-C levels may protect patients from cardiovascular disease [26]. However, recent studies found that in CKD patients, HDL-C had altered structure and became pathogenetic [27, 28]. Dysfunctional HDL-C led to endothelial injury [28], whether they exert deleterious effects on tubular epithelial cells was unclear and requires further study. Altogether, tubular cells are susceptible to lipid disorders. Our study indicated that dysregulated lipid metabolism increased with tubular damage in DN. But the use of statins had a limited effect on the alleviation of lipid disorders. Novel drugs that able to remove ectopic lipid deposition in renal tubules might alleviate tubular damage.

To assess the prognostic value, urinary tubular markers, urinary total protein, urinary albumin, urinary IgG and kidney function were included in a multivariate Cox model. And urinary RBP remained significant as an independent risk factor for ESRD. In nomogram, a conventional model including SCr and total urinary protein was first constructed. Further adding urinary RBP to the model, the prediction ability measured by C-index improved. These results suggested that urinary RBP independently predicted renal prognosis in DN, and might be a useful noninvasive indicator for *primary tubular injury*. Two studies of diabetic patients with macroalbuminuria and all levels of albuminuria also identified urinary RBP as an independent relevant biomarker for kidney disease progression [9, 29]. Treatment targeting proximal tubular cells would benefit diabetic patients with CKD, as clinical trials of sodium-glucose cotransporter 2 (SGLT2) inhibitors could reduce the risk of renal failure [30–32]. Urinary RBP might be a good monitor for therapeutic management of DN and diabetic kidney disease.

The main strength of the study is its longitudinal design allowing assessment of the predictive value of the tubular markers. Besides, patients were biopsy-proven DN, help look into the pathological relationship of the biomarkers. The study also has limitations. It was a retrospective investigation from a single center. But our results showed agreements with those of previous studies, and complemented the prognostic role of urinary RBP in DN. Plus, the tubular injury markers we evaluated reflected a limited aspect of DN tubular injury.

In conclusion, the tubular injury biomarkers, RBP, *β*2-MG and NAG correlated with the severity of tubulointerstitial damage in DN patients. Among them, urinary RBP was the independent risk factor for ESRD. The pathogenesis of tubular impairment is at least partially independent of glomerular lesions even in DN patients with obvious glomerulopathy. Urinary RBP might be a good monitor for therapeutic strategy targeting renal proximal tubules in DN patients.

## Figures and Tables

**Figure 1:** Flowchart for recruitment. DN, diabetic nephropathy; GN, glomerulonephropathy; CKD, chronic kidney disease; RBP, retinol-binding protein; *β*2-MG, *β*2-microglobulin.

**Figure 2:** Correlations between the pathological features and the urinary tubular injury markers, RBP (a-d), *β*2-MG (e-h) and NAG (i-l). RBP, retinol-binding protein; *β*2-MG, *β*2-microglobulin; NAG, N-acetyl-ß-D-glycosaminidase.

**Figure 3:** Associations of urinary RBP (a), *β*2-MG (b) and NAG (c) levels with risk of ESRD with adjustment for age, gender and BMI using restricted cubic spline regressions. The solid line represents the estimated HR, the shaded area represents the 95% CI derived from restricted cubic spline regressions. ESRD, end stage renal disease; RBP, retinol-binding protein; *β*2-MG, *β*2-microglobulin; NAG, N-acetyl-ß-D-glycosaminidase; BMI, body mass index.

**Figure 4:** Renal survival curves of patients with low and high urinary RBP levels. (a) The survival analysis for all DN patients. (b-c) The survival analysis for patients was stratified by total urine protein. DN, diabetic nephropathy; RBP, retinol-binding protein; UPCR, urinary protein to creatinine ratio.

**Figure 5:** Nomogram for renal survival. RBP, retinol-binding protein. BMI, body mass index.

**Table 1:** Cox regression models for ESRD.

	Model1			Model2			Model3			Multivariate stepwise LR		
	HR	95% CI	*p*	HR	95% CI	*p*	HR	95% CI	*p*	HR	95% CI	*p*
Male	1.38	0.91-2.09	0.125	—	—	**—**	—	—	—	1.75	1.06-2.90	**0.029**
Age, years	0.99	0.96-1.01	0.328	—	—	**—**	—	—	—			
BMI,kg/m^2^	0.93	0.89-0.98	**0.011**	—	—	**—**	—	—	—	0.92	0.87-0.97	**0.010**
SCr mg/dL	2.69	2.01-3.46	**<0.001**	2.76	2.12-3.58	**<0.001**	—	—	—	2.29	1.73-3.04	**<0.001**
UPCR, g/g	1.20	1.14-1.27	**<0.001**	1.24	1.18-1.32	**<0.001**	1.22	1.15-1.29	**<0.001**	1.20	1.12-1.29	**<0.001**
Urinary albumin, g/Mol.Cr	1.00	1.00-1.001	**<0.001**	1.001	1.001-1.001	**<0.001**	1.001	1.001-1.001	**<0.001**			
Urinary IgG, g/Mol.Cr	1.01	1.00-1.01	**<0.001**	1.01	1.003-1.01	**<0.001**	1.005	1.003-1.007	**<0.001**			
Urinary RBP, g/Mol.Cr	1.05	1.03-1.06	**<0.001**	1.05	1.03-1.07	**<0.001**	1.05	1.03-1.0	**<0.001**	1.06	1.03-1.10	**0.001**
Urinary *β*2-MG, g/Mol.Cr	1.17	1.10-1.25	**<0.001**	1.18	1.10-1.27	**<0.001**	1.06	0.98-1.14	0.157			
Urinary NAG, U/Mol.Cr	1.20	1.10-1.30	**<0.001**	1.20	1.09-1.30	**<0.001**	1.22	1.11-1.33	**<0.001**			
Hemoglobulin, mg/dL	0.76	0.69-0.83	**<0.001**	0.75	0.68-0.82	**<0.001**	0.82	0.74-0.91	**0.001**	0.88	0.79-0.98	**0.017**
Total cholesterol, mmol/L	1.13	1.01-1.27	**0.041**	1.19	1.05-1.35	**0.007**	1.19	1.05-1.34	**0.005**			
LDL-C, mmol/L	1.08	0.92-1.26	0.359	1.10	0.94-1.30	0.237	0.13	0.96-1.32	0.141			
HDL-C, mmol/L	1.46	0.96-2.22	0.078	1.34	0.84-2.13	0.225	1.76	1.09-2.84	**0.022**			
Systolic BP, mmHg	1.01	1-1.02	0.042	1.01	1.002-1.02	**0.019**	1.01	1.001-1.02	**0.025**			
Diastolic BP, mmHg	1.01	1-1.03	0.073	1.01	1.00-1.03	0.098	1.01	1.00-1.03	0.116			

Model 1 was a univariate analysis for each indicator. Model 2 was adjusted for gender, age and BMI. Model 3 was adjusted for gender, age, BMI and SCr. Multivariate analysis included age, gender, BMI, SCr, UPCR, urinary microalbumin, urinary IgG, urinary RBP, urinary *β*2-MG, NAG, hemoglobulin, total cholesterol and systolic BP. SCr, Serum creatinine; UPCR, urinary protein to creatinine ratio; RBP, retinol-binding protein; *β*2-MG, *β*2-microglobulin; NAG, N-acetyl-ß-D-glycosaminidase. HDL-C, High-density lipoprotein cholesterol; LDL-C, low-density lipoprotein cholesterol; BP, blood pressure.

**Table 2:** Comparisons between diabetic patients with low and high urinary RBP levels.

	Low RBP (n =152)	High RBP (n =153)	*p*
Male, n (%)	126(82.9)	106(69.3)	**0.007**
Age, years	52.63 ± 10.63	51.71 ± 10.29	0.451
BMI,kg/m^2^	24.76 ± 3.36	24.38 ± 3.44	0.336
Follow up, months	20.50(13.84, 31.59)	24.60(12.88, 37.12)	0.579
Diabetic duration, years	8.58 ± 6.52	8.28 ± 5.90	0.666
Diabetic retinopathy, n/N (%)	72/110(65.5)	80/121(66.1)	1
Systolic BP, mmHg	137.05 ± 15.48	145.2 ± 16.57	**<0.001**
Diastolic BP mmHg	80.24 ± 11.43	83.4 ± 11.68	**0.021**
Hemoglobulin, mg/dL	11.59 ± 2.23	11.01 ± 1.92	**0.015**
HbA1c, %	7.53 ± 1.67	7.76 ± 2.00	0.277
Total cholesterol, mmol/L	4.59 ± 1.42	5.02 ± 1.54	**0.011**
Triglyceride, mmol/L	2.12 ± 1.5	1.99 ± 1.13	0.377
HDL-C, mmol/L	1.03 ± 0.35	1.15 ± 0.39	**0.006**
LDL-C, mmol/L	2.55 ± 1.15	2.91 ± 1.2	**0.006**
VLDL-C, mmol/L	0.96 ± 0.69	0.94 ± 0.55	0.653
Uric acid, *μ*mol/L	397.73 ± 86.28	380.47 ± 94.19	0.119
Serum albumin, g/L	35.88 ± 6.55	31.82 ± 6.16	**<0.001**
SCr, mg/dL	1.53 ± 0.68	1.48 ± 0.70	0.415
eGFR, ml/min/1.73m^2^	60.24 ± 29.14	60.42 ± 25.99	0.948
UPCR, g/g	2.1(0.73, 4.23)	3.92(2.69, 5.82)	**<0.001**
Urinary albumin, g/Mol.Cr	66.79(37.47, 121.93)	353.52(213.65, 604.49)	**<0.001**
Urinary IgG, g/Mol.Cr	11.48(4.8, 22.43)	55.1(27.88, 91.2)	**<0.001**
Urinary *β*2-MG, g/Mol.Cr	0.19(0.06, 0.60)	0.59(0.22, 1.59)	**<0.001**
Urinary NAG, U/Mol.Cr	1.31(0.94, 2.33)	2.39(1.60, 3.83)	**<0.001**
Treatment			
RAAS inhibitor	92(60.5)	101(66.0)	0.343
CCB	106(69.7)	110(71.9)	0.707
Statin	54(35.5)	60(39.2)	0.554
Insulin	94(61.8)	113(73.9)	**0.028**

RBP, retinol-binding protein; BP, blood pressure; HbA1c, Hemoglobin A1c; HDL-C, High-density lipoprotein cholesterol; LDL-C, low-density lipoprotein cholesterol; VLDL-C, very low-density lipoprotein cholesterol; SCr, serum creatinine; eGFR, estimated glomerular filtration rate; UPCR, urinary protein to creatinine ratio; *β*2-MG, *β*2-microglobulin; NAG, N-acetyl-*β*-D-glycosaminidase; RAAS, renin-angiotensin-aldosterone system; CCB, calcium channel blocker.

## Data Availability

The data used to support the findings of the study are included within the article.

## Additional Points

*Clarification.* Part of the study had been presented as a poster in abstract form at the World Congress of Nephrology 2022 [33].
